# A Parallel DNA Algorithm for Solving the Quota Traveling Salesman Problem Based on Biocomputing Model

**DOI:** 10.1155/2022/1450756

**Published:** 2022-08-31

**Authors:** Zhaocai Wang, Xian Wu, Tunhua Wu

**Affiliations:** ^1^College of Information, Shanghai Ocean University, Shanghai 201306, China; ^2^School of Information Engineering, Wenzhou Business College, Wenzhou 325035, China

## Abstract

The quota traveling salesman problem (QTSP) is a variant of the traveling salesman problem (TSP), which is a classical optimization problem. In the QTSP, the salesman visits some of the *n* cities to meet a given sales quota *Q* while having minimized travel costs. In this paper, we develop a DNA algorithm based on Adleman-Lipton model to solve the quota traveling salesman problem. Its time complexity is *O*(*n*^2^+*Q*), which is a significant improvement over previous algorithms with exponential complexity. A coding scheme of element information is pointed out, and a reasonable biological algorithm is raised by using limited conditions, whose feasibility is verified by simulation experiments. The innovation of this study is to propose a polynomial time complexity algorithm to solve the QTSP. This advantage will become more obvious as the problem scale increases compared with the algorithm of exponential computational complexity. The proposed DNA algorithm also has the significant advantages of having a large storage capacity and consuming less energy during the operation. With the maturity of DNA manipulation technology, DNA computing, as one of the parallel biological computing methods, has the potential to solve more complex NP-hard problems.

## 1. Introduction

In the quota traveling salesman problem (QTSP), a traveling salesman can sell a certain number of items in each city, whose request is to visit enough cities to meet a certain sales quota and let him return to the original city. The goal of QTSP is to find the shortest path that could satisfy the requirement of he salesman. That is, the optimal solution for the QTSP is to visit a loop of a certain number of cities, where the weighted sum of the cities visited satisfies a deterministic value and the path weight sum of the loop is minimal. The QTSP was first introduced by Awerbuch et al. in 1995 [1]. And the QTSP has many applications in reality, for example, the route selection of emergency vehicles. With the frequent occurrence of natural disasters, the rescue of emergency vehicles for different areas has attracted people's attention. Due to the different degrees of disasters suffered form different regions, emergency supplies should be reasonably distributed and delivered to the demand point. Emergency vehicles need to carry certain emergency supplies to service the needs of the cities, and return to the starting city. The emergency vehicle receives a weighted map of multiple cities, each of which has an additional requirement to designate the emergency supplies that can be distributed in that city. In this case, the target problem that consumes the least total time can be described by the QTSP.

The QTSP can be considered a special case of the prize collection traveling salesman problem (PCTSP), which was initially presented by Balas [2]. In the PCTSP, a traveling salesman must visit a number of cities, each of which has rewards and penalties associated with it. Whenever a city is visited, he receives the relevant reward, while whenever that city is not visited, there is a corresponding penalty. In addition, there are costs associated with traveling between two cities. The goal is to minimise the sum of the travel costs and the penalties paid, while ensuring that the minimum prize is received. If the penalties of the cities are regarded as zero, PCTSP evolves into QTSP. In 2008, Ausiello et al. [3] analyzed the online version of the PCTSP and presented the corresponding algorithm. They give a 7/3 competitive algorithm, compared to a lower bound of 2 on the competitive ratio of any deterministic algorithm, and combined the method with an approximation algorithm to obtain an *O*(1)-competitive algorithm that run in polynomial time. In 2013, Pedro et al. [4] proposed a simple but effective tabu search method to solve PCTSP, which improved several upper bounds for the instances considered. If the assigned quota is zero, the QTSP degenerates into a traditional online traveling salesman problem (OLTSP), in which traveling salesman does not know in advance information about demand, but will be aware of them while traveling. For example, fast food delivery, item pickup and so on. Ausiello [5] proposed OLTSP algorithm, studied their competitive ratio, and compared it with the optimal solution to the corresponding offline problem. They discuss OLTSP in two separate categories. The first is where the server is not required to return to the origin node after all submitted requests have been delivered. For this problem, the paper gave a 2.5 competing algorithm for a class of metric spaces and a 7/3 competing algorithm for the real line. For an alternative version of the problem that requires a return to the origin node, they gave the optimal 2-competition algorithm for the above general class of metric spaces.

In the QTSP, if each city has a weight of one, the situation becomes a problem of finding the minimum tour to visit *k* cities in a given graph, which is related to the *k*-Minimum Spanning Tree (*k*-MST) problem. Given an undirected graph with non-negative edge weights on *n* nodes and an integer *k* ≤ *n*, the goal is to find the tree with the smallest weight that spans *k* vertices. Garg [6] showed that a 3-approximation algorithm for the *k*-MST problem can be implemented using a variant form. He also showed that the completeness gap of the natural integer programming formulation of the *k*-MST problem is also three, suggesting that a different approach may be needed to further improve the performance ratio of the *k*-MST problem. In 1998, Awerbuch et al. [7] solved the *k*-MST problem by providing a log^2^(*k*) approximation to improve on the previous best bound of $O\left(\sqrt{k}\right)$. In 1999, Blum [8] proposed a bicriteria approximation algorithm to improves efficiency by a factor of 17 for the *k*-MST with *n* nodes, whose time complexity was *O*((*n*^2^)log^2^(*n*)). The main subroutine of the algorithm was an approximate algorithm by Goemans and Williamson for solving the prize-collecting Steiner tree problem.

Due to the wide applicability of QTSP, the problem has gradually received the attention of research scholars [9]. A further development of the QTSP study is to combine release time with vertices, where the city *v* can only be visited at or after the release time and the salesman can travel at most at unit speed, with the goal of finding a city subset *V*′ that reach the quota *Q* and travel on *V*′ to minimise the completion time, i.e. the time for the salesman to visit all cities in *V*′ and return to the origin node. QTSP is generally divided into two categories: online QTSP and offline QTSP [10]. A QTSP with release times is called an offline QTSP if the release times, weights and positions of the cities are already known before the salesman departs. However, in many cases, all information is assumed and holds completely a priori, from which an online QTSP is derived. In an online QTSP, each city *v* appears at its release time *r*_*v*_, but the release times, weights and even the existence of the cities are only known after its appearance is known. In 2004, Ausiello et al. [11] presented the lower bounds of the online QTSP under the general metric space and the corresponding competitive algorithm, and analyzed the situation where the metric space was half line. In 2014, Yu et al. [12] analyzed the QTSP of four variants based on the symmetry of the measurement. Then they proposed the optimal deterministic algorithm for each variant defined on a general space, a half line, or a real line. In 2020, Silva et al. [13] proposed a mathematical formula and heuristic algorithm based on ant colony optimization for the variant of the QTSP: Quota Traveling Salesman Problem with Passengers, Incomplete Ride and Collection Time (QTSP-PIC). In the QTSP-PIC, the salesman is the driver of the vehicle. Since the trip is pre-arranged, passengers can request a ride and reduce the cost of the trip by splitting the fare with the driver. However, up to now, no algorithm has been proposed for the offline QTSP problem. On the other hand, QTSP has proven to be an NP-hard problem and its pursuit of efficient algorithms has been a hot topic of interest for many scholars [7, 13]. In this paper, we attempt to solve the problem in polynomial time using a new intelligent algorithm (DNA algorithm) to significantly reduce the computational complexity of this NP-hard problem.

The remaining of the paper is organized as follows: Section 2 introduces the relevant background in detail, including the Adleman-Lipton model and QTSP.  Section 3 comes up with the DNA algorithm to figure out the QTSP and analyzes the feasibility and performance of the algorithm. In Section 4, experimental results of simulated DNA calculation are presented. Finally, we come to the conclusion and prospects the future researched work.

## 2. Background Knowledge

This section is divided into three sub-sections, introducing the biological knowledge and the development of DNA computing, explaining the Adelman-Lipton model and describing the QTSP.

### 2.1. Development of DNA Computing Technology

Biological computing is a new type of molecular biocomputing method based on DNA molecules and related enzymes, which uses biochemical reactions to calculate DNA strands. Biological computing pioneers a new way of algorithms [14, 15]. Due to the natural characteristics of DNA molecules, such as specificity, high parallelism and microfineness, molecules can be stored in high capacity and manipulated in parallel. It makes DNA computing has significant advantages, such as very fast computing speed, tremendous storage capacity, and less energy consumption during computing, which also has strong applicability and is widely used to solve NP-hard problems, such as the 0–1 integer programming problem, the satisfiable (SAT) problem, and so on.

In 1994, Adleman [16] successfully solved the Hamiltonian path problem (HPP) in test tubes by dealing with DNA strands. Lipton [17] proved that Adleman technology can be used to solve the SAT problem. Since then, many researchers have used the DNA computing to solve various problems. Ouyang et al. [18] studied a method using molecular biology technology to solve the maximal clique problem, mapping the set to the binary numbers, and then removing and classifying them. The success of the experiment provided stronger evidence for solving complex problem using DNA computing later. Narayanan and Spiridon [19] extended Adelman and Lipton's basic DNA algorithm technique by proposing a method for representing simple arc information, that is, distances between cities in a simple map. This method, while dealing with distances, could also be used with appropriate modifications and extensions to deal with arc labels in general. In 1998, Smith et al. [20] solved the SAT problem based on surface-based DNA model, which allowed a much wider scope for DNA computing to be played out. Chang and Guo [21] proved that basic biological operations can solve the set cover problem, and further presented the cover problem by 3-sets. Guo et al. [22] solved the dominating-set problem by using stickers to build a solution space for DNA molecules. Chang et al. [23, 24] solved the independent set problem and the vertex cover problem, using the super computer model based on DNA and the quantum algorithm combined with DNA computing, respectively. Wang et al. [25] used the proposed DNA algorithm to realize the task scheduling problem with *O*(*n*^2^) time complexity. Lee et al. [26] presented a biased molecular algorithm based on the thermodynamic properties of DNA and a numerical representation of the encoding by designing the variation of the melting temperature of the DNA strands. The method has been successfully applied to traveling salesman problems on weighted graphs. Unlike other DNA computational methods that focus on solving logical problems, this work extends the capabilities of DNA computation to solving numerical optimization problems and clearly represents a significant advance. In contrast, Wang et al. [27] also used DNA biological manipulation to complete the determination and search for the optimal solution to the traveling salesman problem. The difference is that in characterising the length of the path between cities, weight information is added to the initial strand to simplify later operations. In 2016, Sanches and Soma [28] solved two NP-hard problems for DNA computing given biological operations, two of which are minimization of open stacks and matrix bandwidth minimization. In 2018, Inrahim et al. [29] proposed an improved evolutionary DNA technology based on conventional DNA technology to solve job scheduling problem. In 2019, Wang et al. [30] designed a bio-inspired computing model to solve the capacitated vehicle routing problem. In 2020, Tian et al. [31] showed a DNA algorithm with *O*(*n*^2^) time complexity for the job shop scheduling problem. For the generalised traveling salesman problem (GTSP), Ren et al. [32] used DNA biological chains to represent different vertices, point groups and weights, and found the optimal solution of the problem using a series of different DNA sequence biochemical reactions. The feasibility of the algorithm is demonstrated while reducing the time complexity to *O*(*n*^2^). Zhong et al. [33] proposed DNA computing inspired networks design (DNAND) for high-performance deep network automatic learning. DNA computing has been combined with various control technologies, forming DNA computing models based on chains displacement, DNA computation based on ribozyme, DNA computation based on surface, DNA computation based on nanoparticles, and so on [34–36].

### 2.2. The Adleman-Lipton Model

DNA, whose basic unit is deoxyribonucleic acid, is a polymer compound. Each molecule of deoxyribonucleic acid is composed of one molecule of phosphoric acid, one molecule of deoxyribose, and one molecule of nucleobase. The bases of different nucleotides interact to form hydrogen bonds, in which adenine (*A*) pairs with thymine (*T*), and guanine (*G*) pairs with cytosine (*C*). Hence, DNA can form a rotating double helix structure from a long single strand (Figure 1). Since base pairs can arrange repeatedly, DNA molecules have diversity.

The process of DNA computing is to map the problems into DNA molecular chains, and use the principle of complementarity to generate various data pools under the action of biological enzymes. Then, the constraints of the problems are mapped to the controlled biochemical reaction process of the DNA chains in a highly parallel way. Finally, the detection methods, such as polymer chain reaction (PCR), probes, electrophoresis and so on, are used to obtain the calculation results we need. The above processes are also the logical courses of DNA computing and Adleman-Lipton model [37]. The core problem is to take the encoded DNA strands as input, and complete biological calculations through test tubes methods, surface methods, etc., to obtain all the solution spaces. In DNA computing, the length of a single strand of DNA is is determined by the number of nucleotides that make up that single strand. Thus, if a single-stranded DNA contains 10 nucleotides, the length of the strand is considered to be 10 and is called 10 mer.

Suppose that a set of DNA strands (single strands) in a test tube, it is a collection of finite strings composed of the alphabets *A*, *G*, *C*, *T*. Some biological experiments can be performed on the test tube. The specific operations can be described as follows:

1. Merge (*T*_1_, *T*_2_): Given two test tubes *T*_1_ and *T*_2_, the operation is to mix the two test tubes in tube *T*_1_, and the tube *T*_2_ is empty;
2. Denaturation (*T*): Given a test tube *T*, the operation is to separate all double strands of DNA in test tube *T* into two corresponding single strands;
3. Annealing (*T*): Given a test tube *T*, the operation is to generate all possible double strands from the single-stranded DNA in the test tube *T* according to the Watson-Crick base pairing principle [38], and still store them in *T* after annealing;
4. Separation (*T*_1_, *x*, *T*_2_): Given two test tubes *T*_1_, *T*_2_ and a single DNA strand *x*, the operation is to remove all DNA single strands containing *x* from the tube *T*_1_, and put all DNA single strands containing *x* into the test tube *T*_2_;
5. Discard (*T*): Given a test tube *T*, the operation is to remove all strands in the test tube *T*;
6. Append-head (*T*, *s*): Given a test tube *T* and DNA strands with specific code *s*, the operation is to attach DNA strands *s* to the head of each strand in the tube *T*;
7. Append-tail (*T*, *s*): Given a test tube *T* and DNA strands with specific code *s*, the operation is to attach DNA strands *s* to the end of each strand in the tube *T*;
8. Selection (*T*_1_, *L*, *T*_2_): Given two test tubes *T*_1_, *T*_2_ and an integer *L*, the operation is to move all DNA strands of *L*-length from tube *T*_1_ to test tube *T*_2_, and the rest of the DNA strands are still in the test tube *T*_1_;
9. Cutting (*T*, *ω*_1_*ω*_2_): Given a test tube *T* and strings with specific code *ω*_1_*ω*_2_, the operation is to cut every strand containing [*ω*_1_*ω*_2_] in tube *T* into different strands from the middle, that is [⋯*ω*_1_*ω*_2_⋯]⟶[⋯*ω*_1_], [*ω*_2_⋯].
10. Sort: Given test tubes (HTML translation failed), *T*_2_ and *T*_3_, the operation is to move the shortest and the longest DNA strands to test tube *T*_2_ and *T*_3_, respectively, while the rest of the DNA strands are still in the test tube;
11. Read (*T*): Given a test tube *T*, the operation is to identify the composition of biological strands in the tube *T*.

All of the above operations can be achieved in certain biological steps. In previous studies, many researchers reasonably assumed that the complexity of each operation was *O*(1) to analyze different problems [34, 35, 39–41]. The research in this paper also uses these operations to implement the algorithm of QTSP.

### 2.3. Quota Traveling Salesman Problem

The QTSP is defined on a graph *G*=(*V*, *A*), where *V* is the set of *n* nodes and *A* is the set of *m* edges. Each node *i*(*i* ∈ *V*) has a corresponding weight *w*_*i*_ and each edge (*i*, *j*)((*i*, *j*) ∈ *A*) has a corresponding distance value *d*_*ij*_. The minimum amount of quota to be collected is given by *Q*. The QTSP is to find the shortest cycle satisfying quota *Q* in *G* , where the path starts from and returns to the origin. This paper mainly studies symmetric offline QTSP. The formulation defines the binary variable *x*_*ij*_ ∈ {0,1}, if the edge is passed in the route, then *x*_*ij*_ is equal to one; otherwise it is 0. In addition, it also requires *y*_*i*_ ∈ {0,1}, if vertex *i* is visited, *y*_*i*_=1, otherwise *y*_*i*_=0. Moreover, continuous variables *f*_*ij*_ ≥ 0 is used to prevent sub-routing. The mixed-integer programming formulation of the QTSP can be given as follows [42]:

(1) $$\begin{array}{c} min\;Z=\sum_{\left(i,j\right)\in A}d_{ij}x_{ij}, \end{array}$$

(2) $$\begin{array}{c} \mathrm{s.}t.:\sum_{\left(i,j\right)\in A}x_{ij}=y_{i}\;\forall i\in V, \end{array}$$

(3) $$\begin{array}{c} \sum_{\left(i,j\right)\in A}x_{ij}=y_{j}\;\forall j\in V, \end{array}$$

(4) $$\begin{array}{c} \sum_{i\in V}w_{i}y_{i}\geq Q, \end{array}$$

(5) $$\begin{array}{c} \sum_{\left(j,i\right)\in A}f_{ji}-\sum_{\left(i,j\right)\in A}f_{ij}=y_{i}\;\forall i\in V, \end{array}$$

(6) $$\begin{array}{c} f_{ij}\leq \left(n-1\right)x_{ij},\;\forall \left(i,j\right)\in A, \end{array}$$

(7) $$\begin{array}{c} x_{ij}\in \left\{0,1\right\},\;\forall \left(i,j\right)\in A, \end{array}$$

(8) $$\begin{array}{c} y_{i}\in \left\{0,1\right\},\;\forall i\in V, \end{array}$$

(9) $$\begin{array}{c} f_{ij}\geq 0,\;\forall \left(i,j\right)\in A. \end{array}$$

The objective function (1) minimises the travel cost. Constraints (2) and (3) guarantee that the salesmen visit and leave node *i* accurately. Constraint (4) ensures that the salesman gets at least the minimum quota through different vertices. Constraints (5), (6) and (9) void the existence of sub-tours. Constraints (7) and (8) are used to indicate whether edges and vertices in the graph are visited by the salesmen.

Given a complete graph with six cities, Figure 2 illustrates an instance of QTSP. Starting from *v*_1_, the salesman can go to any city. The edge weights in the graph correspond to the distance between cities, while the vertex weights in the graph correspond to the quota of cities. The salesman needs to only visit other cities once for starting from *v*_1_, and the tour is the shortest one that meet the minimum quota *Q*. In this case, the salesman quota requirement is 7. He starts at point *v*_1_, and goes through the cities, such that the sum of the city weights is equal to 7 or greater than 7.

After logical calculations, the shortest cycle that meets the requirements is:

(10) $$\begin{array}{c} v_{1}⟶v_{2}⟶v_{5}⟶v_{3}⟶v_{1}. \end{array}$$

We can conclude that the sum of the weights in the shortest cycle is 9. In the small-scale data problem, we can easily get the optimal solution of the problem. However, as the scale of the problem continues to expand, it will become more and more difficult. Therefore, it is eager to have a new algorithm to solve it efficiently.

## 3. A DNA Algorithm for the Quota Traveling Salesman Problem

This section starts with the preliminary thought and then gives the coding scheme of the proposed algorithm. The detailed algorithm is finally presented.

### 3.1. Preliminary Thought

As described earlier, DNA computing solves the optimal path problem in three stages: mapping information to DNA strands, selecting all possible path strands and reading the optimal solution strand [43]. Among them, the DNA encoding of the information is very essential, because the quality of the encoding determines the complexity of the subsequent operations and affects the accuracy of the experiment [44, 45]. When selecting all possible path strands, the original DNA strands are screened according to the constraints of the specific problem. After eliminating the DNA strands that do not satisfy all constraints, the last remaining ones are the DNA strands corresponding to feasible solutions to the problem. This aspect is the core of DNA computing and plays a key role in the accurate solution of the problem [46, 47]. Taking QTSP as an example, since the feasible solution of the problem is a loop tour that starts from the origin node and returns it after passing through a series of vertices at most once, and the sum of the weights of the loop tour vertices is required to be no less than *Q*. Therefore, the path strands that pass through a vertex many times or do not satisfy the weight constraint are eliminated. Meanwhile, to eliminate the influence of the loop tour passing through different numbers of vertices on the strands length, an auxiliary chain of the same length is added to the vertices not passed in the loop tour for the optimal solution selection. Finally, after adding the path weight chains on the loop tour, the shortest length DNA strands mean the minimum sum of path weights. The optimal solution of the QTSP is obtained by reading its encoding information.

Specifically, the steps of the DNA algorithm for the QTSP are as follows:

**Step 1 .**

Generate the initial solution of all paths, starting from the origin node *v*_1_ and ending at the node *v*_1_;

**Step 2 .**

According to different constraints, perform operations to obtain feasible solutions;

**Step 3 .**

Attach the weight value of each route passing node to filter out the routes that meet the quota;

**Step 4 .**

Add the tail to the end of the feasible strands, which represents the weights of the passing edge;

**Step 5 .**

Sort the feasible solutions and read the optimal results of the quota traveling salesman problem.

Figure 3 shows the algorithm flow chart. According to the flow chart, the steps of the algorithm can be clearly understood.

### 3.2. Notations and Symbols

In order to standardise and facilitate the expression and understanding of the algorithm, the definition and description of the notations and symbols used in the paper are given in Table 1.

### 3.3. Encoding

Effective coding is the key to mapping practical problems to computational models of DNA molecules. The symbols *A*_*i*_, *B*_*i*_ (*i* ∈ {1,2,…, *n*}) used to represent a part of the vertex strands, and then the connected symbol *A*_*i*_*B*_*i*_ used to represent the DNA strands of vertex *v*_*i*_, assuming that the length of each symbol is *t* mer. The symbol # indicates the ends of the DNA strands. Simultaneously, the DNA strands need to be connected to form double strands with the help of complementary strands $\bar{B_{i}A_{j}}\;\left(\left(i,j\right)\in E\right)$. Obviously, the length of the DNA strands is largely affected by the size of the involved problem. Furthermore, to distinguish different routes strands, chains *Y* is designed whose length is *t* mer. At the same time, in order to calculate the weights of the nodes and edges, the corresponding biological chains *ψ* and *X* of length *t*-mer are designed.

### 3.4. Detailed DNA Algorithm

For a QTSP with *n* nodes, we generate DNA strands to represent different traveling salesman routes. The initial test tubes are:

(11) $$\begin{array}{c} T_{1}=\left\{\#A_{1}B_{1},A_{2}B_{2},\ldots ,A_{n}B_{n},A_{1}B_{1}\#\right\},\\ T_{2}=\left\{\bar{B_{i}A_{j}}|\left(i,j\right)\in E,i\neq j\right\}. \end{array}$$

Taking the problem in Figure 2 as an example, the test tubes:

(12) $$\begin{array}{c} T_{1}=\left\{\#A_{1}B_{1},A_{2}B_{2},A_{3}B_{3},A_{4}B_{4},A_{5}B_{5},A_{6}B_{6},A_{1}B_{1}\#\right\},\\ T_{2}=\left\{\bar{B_{1}A_{2}},\bar{B_{1}A_{3}},\bar{B_{1}A_{4}},\bar{B_{1}A_{5}},\bar{B_{1}A_{6}},\bar{B_{2}A_{1}},\bar{B_{2}A_{3}},\bar{B_{2}A_{4}},\bar{B_{2}A_{5}},\bar{B_{2}A_{6}}\right),\\ \bar{B_{3}A_{1}},\bar{B_{3}A_{2}},\bar{B_{3}A_{4}},\bar{B_{3}A_{5}},\bar{B_{3}A_{6}},\bar{B_{4}A_{1}},\bar{B_{4}A_{2}},\bar{B_{4}A_{3}},\bar{B_{4}A_{5}},\bar{B_{4}A_{6},}\\ \left(\bar{B_{5}A_{1}},\bar{B_{5}A_{2}},\bar{B_{5}A_{3}},\bar{B_{5}A_{4}},\bar{B_{5}A_{6}},\bar{B_{6}A_{1}},\bar{B_{6}A_{2}},\bar{B_{6}A_{3}},\bar{B_{6}A_{4}},\bar{B_{6}A_{5}}\right\}. \end{array}$$

Each execution of steps (1), (2) and (3) forms a legal or illegal travel route for elements representing different vertices in *T*_1_ and *T*_2_. Next, step (4) and step (6), respectively, filter out sets that start the route with *v*_1_ and those that end the route at *v*_1_ from the set. Now, the set stored in *T*_4_ represents the traveler's path that starts and ends at a fixed vertex *v*_1_. After the execution of the above Algorithm 1, all the DNA strands of the path starting from *v*_1_ to are obtained in the tube *T*_4_. In the example of Figure 2, the strands #*A*_1_*B*_1_*A*_4_*B*_4_*A*_5_*B*_5_*A*_1_*B*_1_# representing the route *v*_1_⟶*v*_4_⟶*v*_5_⟶*v*_1_ is generated in *T*_4_.

In this way, it can be obtained all possible path chains of the QTSP in the test tube. Namely, the test tube is the data pool. Since each of the above operations perform in time *O*(1) [34, 35, 39–41], Algorithm 1 can be completed in time *O*(1).

Each execution of step (1) stores the travel route through the city representing “*v*_*j*_” into *T*_5_. Each time step (2) is performed, and then *YY* is appended to the end of the route that does not pass through the -city. Next, execution of step (3) merges the two tubes *T*_4_ and *T*_5_. After repeating steps (1) through (4), all *n* elements are inspected. Then, step (5) will filter out the DNA strands in the tube *T*_4_ in the length of (2*n*+4)*t*. A feasible path that does not go through a vertex supplements its length by appending DNA strands of the same length. In the QTSP, each vertex is required to be delivered only once by the salesman. In order to eliminate the distress of decision making caused by the different number of cities visited in the tour, determine in turn whether the city *v*_*j*_ has been visited in the tour, if so, the chains *A*_*j*_*B*_*j*_ are included in the strands, otherwise, it should add the auxiliary chain *YY* and ‖*A*_*j*_*B*_*j*_‖=‖*YY*‖ to eliminate the influence of the number of cities on the strands length. After adding the tail chains *YY*, if the DNA strands exceed a certain length, it indicates that the route passes through a vertex many times, so the infeasible strands are discarded. For example, after the Algorithm 2, the route *v*_1_⟶*v*_4_⟶*v*_5_⟶*v*_1_ in Figure 2 is represented by DNA strands #*A*_1_*B*_1_*A*_4_*B*_4_*A*_5_*B*_5_*A*_1_*B*_1_#*YYYYYY*.

The operation uses a “For” clause, so the Algorithm 2 can be done in time *O*(*n*), as each of the above operations was done in time *O*(1).

Each execution of steps (1) and (2) appends the vertex weights (‖*ψ* ⋯ *ψ*‖=*w*_*j*_) at the head of the strands, if this route passes the *j*-city. The number of *ψ* is related to vertex weights *w*_*j*_. After repeated steps (1) through (4), the length of the DNA strands in the tube *T*_6_ is related to the weights that passes through the vertices. Steps (5) and (6) discard illegal DNA strands whose travel path quota is less than *Q*. Step (7) cuts and discards the additional *ψ* ⋯ *ψ* in the legal DNA strands.

For example, after the step (4), the route *v*_1_⟶*v*_3_⟶*v*_4_⟶*v*_5_⟶*v*_1_ in Figure 2 is represented by DNA strands

(13) $$\begin{array}{c} L_{1}=\underset{W_{3}=3}{\underset{︸}{\psi \psi \psi }}\underset{W_{4}=2}{\underset{︸}{\psi \psi }}\underset{W_{5}=2}{\underset{︸}{\psi \psi }}\underset{2\times 6+4}{\underset{︸}{\#A_{1}B_{1}A_{3}B_{3}A_{4}B_{4}A_{5}B_{5}A_{1}B_{1}\#YYYY}}. \end{array}$$

Since the sum of vertex weights of the strands *L*_1_ is not less than *Q*(3+2+2 ≤ 7), they are still retained in tube (HTML translation failed) after step (7). Corresponding to this, DNA strands $L_{2}=\underset{W_{4}=2}{\underset{︸}{\psi \psi }}\underset{W_{5}=2}{\underset{︸}{\psi \psi }}\underset{2\times 6+4}{\underset{︸}{\#A_{1}B_{1}A_{4}B_{4}A_{5}B_{5}A_{1}B_{1}\#YYYYYY}}$ representing the route *v*_1_⟶*v*_4_⟶*v*_5_⟶*v*_1_ should be eliminated because it does not meet the quota constraint (2+2 < 7).

Next, in order to eliminate the influence of vertex weight value on the shortest route selection, after selecting the feasible route strands, we divide and remove the weight chains of vertices from the feasible ones. For example, strands *L*_1_ is cut to *ψψψψψψψ* and #*A*_1_*B*_1_*A*_3_*B*_3_*A*_4_*B*_4_*A*_5_*B*_5_*A*_1_*B*_1_#*YYYY* by step (7). Then, is selected to be stored in the tube *T*_9_ by step (8).

This operation uses the “For” clause twice in sequence, so the Algorithm 3 can be completed in time *O*(*n*^2^).

Algorithm 4 is a nested loop, where the loop index variables *i* and *j* range from 1 to *n*. Each execution of step (1) stores the DNA strands passing through the edge (*i*, *j*) from the tube *T*_9_ to the *T*_10_. If the tube *T*_10_ is not empty, step (2) appends DNA chains *XX* ⋯ *X* to the end of the DNA strands representing the routes passing through the edge (*i*, *j*), where the number of *X* equals to the weight of the edge (*i*, *j*). The step (3) merges the treated *T*_9_ and *T*_10_ tubes. The execution of step (4) indicates that *T*_10_ is empty and the next loop continues. After repeated execution (1) to (5), the length of the DNA strands stored in the *T*_9_ is related to the edge weights of the travel routes. Taking the route (*v*_1_⟶*v*_2_⟶*v*_3_⟶*v*_5_⟶*v*_1_) in Figure 2 as an example, the corresponding DNA strands is:

(14) $$\begin{array}{c} \#A_{1}B_{1}A_{2}B_{2}A_{3}B_{3}A_{5}B_{5}A_{1}B_{1}\#YYYY\underset{d_{12}}{\underset{︸}{X}}\underset{d_{23}}{\underset{︸}{X}}\underset{d_{35}}{\underset{︸}{XX}}\underset{d_{51}}{\underset{︸}{XXXXXXXX}} \end{array}$$

The weight of the route above adds up to 11 (*d*_12_+*d*_23_+*d*_35_+*d*_51_=11).

And the operation also uses two “For” nested clauses, thus the Algorithm 4 can be done in time *O*(*n*^2^).

Among many different routes, the best solution of the QTSP has the smallest weight value. We search for the shortest DNA strand in the test tube *T*_9_, which represents the optimal solution of the problem. Each execution of steps (1) and (2) selects the longest and shortest DNA strands and reads the shortest DNA strands, then the algorithm terminates. Obviously, the Algorithm 5 works in time *O*(1).

### 3.5. The Correctness and Complexity of the Proposed Algorithm

The following theorems are used to describe the time complexity, the number of the tubes used and the length limit of the library strands in solution space for the DNA algorithm.

**Theorem 1 .**

The DNA algorithm of the QTSP has *O*(*n*^2^+*Q*) time complexity and uses *O*(*n*^2^) tubes based on the Adleman-Lipton model.

**Proof**

The algorithm mainly includes four steps. Algorithm 1 is mainly used to determine the set of chains starting and ending from a particular vertex, and remove any illegal chains from all possible library chains. Algorithm 1 takes one “Merge” operation, one “Annealing” operation, two “Separation” operations and two “Discard” operations. Next, at most (*n* − 1) adjacent vertices are filtered. Algorithm 2 takes (*n* − 1) “Separation” operations, (*n* − 1) “Append-tail” operations, (*n* − 1) “Merge” operations and one “Selection” operation. On the Algorithm 3 of step (1) through step (4) is used to calculate the weight value of each vertex, and takes (*n* − 1) “Separation” operations, (*n* − 1) “Merge” operations and (*n* − 1) “Append-head” operations. Next, step (5) and step (6) take (*Q* − 1) “Selection” operations and (*Q* − 1) “Discard” operations. Starting from Algorithm 4, (*n* × *n*) “Separation” operations are carried out, with no more than *n* × *n* “Append-tail” operations, “Merge” operations and “Discard” operations. Algorithm 5 takes at most one “Sort” operation and one “Read” operation. Therefore, from the above statement, we can immediately infer that in the Adleman-Lipton model, the solutions of the QTSP has an *O*(*n*^2^+*Q*) biological operations. Meanwhile, we have no more than the (*n* × *n*+2 × *n*+*Q*+5) tubes are used. Therefore, it can be immediately inferred from the above statement that QTSP with *n* vertices and *Q* quota requirements is solved using *O*(*n*^2^+*Q*) biological manipulation and *O*(*n*^2^) test tubes.

The DNA algorithm time complexity *T* is as follows:

(15) $$\begin{array}{c} T\left(\text{Algorithm }1\right)=O\left(7\right)=O\left(1\right);\\ T\left(\text{Algorithm }2\right)=O\left(4\left(n-1\right)+1\right)=O\left(n\right);\\ T\left(\text{Algorithm }3\right)=O\left(4\left(n-1\right)+2\left(Q-1\right)+2\right)=O\left(n+Q\right);\\ T\left(\text{Algorithm }4\right)=O\left(4nn\right)=O\left(n^{2}\right);\\ T\left(\text{Algorithm }5\right)=O\left(2\right)=O\left(1\right);\\ T=T\left(\text{Algorithm }1\right)+T\left(\text{Algorithm }2\right)+T\left(\text{Algorithm }3\right)\\ +T\left(\text{Algorithm }4\right)+T\left(\text{Algorithm }5\right)\\ =O\left(1\right)+O\left(n\right)+O\left(n+Q\right)+O\left(n^{2}\right)+O\left(1\right)\\ =O\left(n^{2}+Q\right). \end{array}$$

**Theorem 2 .**

The result chains of the QTSP can be searched within a limited length range.

**Proof**

Set *l*=∑∑(*i*, *j*) and the length of the different strands is:

(16) $$\begin{array}{c} \left\|A_{k}\right\|=\left\|B_{k}\right\|=\left\|\#\right\|=\left\|Y\right\|=\left\|X\right\|=\left\|\psi \right\|=t\text{ mer }k\in \left\{1,2,\ldots ,n\right\} \end{array}$$

The length of DNA strands *L* corresponding to the optimal scheduling in Algorithm 5 is:

(17) $$\begin{array}{c} \#A_{1}B_{1}A_{k_{1}}B_{k_{1}}A_{k_{2}}B_{k_{2}}\cdots A_{k_{r}}B_{k_{r}}A_{1}B_{1}\#YY\cdots Y\underset{p}{\underset{︸}{XX\cdots X}} \end{array}$$

When edge (*i*, *j*) chain is included in the routing strands, we add *XX* ⋯ *X* with *d*_*ij*_ length. The number *p* represents the number of *X*. Therefore, we can reasonably infer that the length of the DNA strand is:

(18) $$\begin{array}{c} \left\|L\right\|=\left\|\#\right\|+\left\|A_{1}\right\|+\left\|B_{1}\right\|+\left\|A_{k_{1}}\right\|+\left\|B_{k_{1}}\right\|+\left\|A_{k_{2}}\right\|+\left\|B_{k_{2}}\right\|+\cdots +\left\|A_{k_{r}}\right\|\\ +\left\|B_{k_{r}}\right\|+\left\|A_{1}\right\|+\left\|B_{1}\right\|+\left\|\#\right\|+\left\|Y\right\|+\cdots +\left\|Y\right\|+\left\|X\right\|+\cdots +\left\|X\right\|\\ =2\left\|\#\right\|+2\left\|A_{1}\right\|+2\left\|B_{1}\right\|+\underset{2r}{\underset{︸}{\left\|A_{k_{1}}\right\|+\left\|B_{k_{1}}\right\|+\cdots +\left\|A_{k_{r}}\right\|+\left\|B_{k_{r}}\right\|}}\\ +\underset{2\left(n-r-1\right)}{\underset{︸}{\left\|Y\right\|+\cdots +\left\|Y\right\|}}+\underset{p}{\underset{︸}{\left\|X\right\|+\cdots +\left\|X\right\|}}\\ =\left(2n+4\right)t+pt\\ ∵0\leq p\leq l\\ ∴\left(2n+4\right)t\leq \left\|L\right\|\leq \left(2n+4\right)t+lt. \end{array}$$

Hence, we get the solution within a certain chain length.

## 4. Simulation Experiment of DNA Algorithm

DNA computing relies on the biochemical reactions of DNA molecules, which can lead to incorrect or unwanted calculations due to their technical difficulties. Since the accuracy of DNA computing directly affects the results, the information representation of each symbol in the question plays a decisive role. Otherwise, it will lead to the accumulation and diffusion of errors in the biochemical reaction. Therefore, it is necessary to design DNA sequences suitable for simulation experiments. A Python program was designed to perform the simulation experiments, and the similar approach have been used in previous studies [48]. The computer used for the simulations has an AMD Ryzen 7 PRO 4750U processor with a clock speed of 1.70 GHz, Windows 10, 64 bit and 16G of RAM. It is difficult to find the set of instances for the offline QTSP so that we generated the instances of the QTSP through the PCTSP instances. The following conditions are adopted to generate the instances based on the characteristics of the PCTSP and the correlation between them.

- Eliminate penalty mechanism in the PCTSP, that is, the penalties *γ*_*i*_  = 0.
- Calculate the rated quota *Q* using the formula *σ*∑_*i*=1_^*n*^*p*_*i*_ with *σ* ∈ {0.2, 0.5, 0.8}.

The PCTSP instance names are supplemented to name the QTSP instances in order to distinguish and identify the instances. The decimal parts of the sigma values are intercepted to indicate different cases, and they are spliced to the end of the PCTSP instance name to distinguish between instances. An example is presented in Table 2 to present the naming convention more clearly [49].

Based on the above rules, the instance generator are designed to create the data files. Then, some of the instances are selected to be solved with the solver we designed and the corresponding results are obtained. The basic information from 64 instances addressed by the solver are summarized in Table 3 and the routes are presented in Table 4. In Table 3, Id represents the serial number of the instance, *n* represents the total number of nodes in the instance, *Q* represents the minimum amount, *Q*_*r*_ and *D*_*r*_ denote the sum of quotas and the sum of weights of the resultant router, respectively. Time indicates the time cost (in seconds) consumed by the instance to be solved by the solver.

Routes can be obtained by decoding the DNA strands, and examples can be given to understand more clearly the process of solving examples of DNA algorithms. Taking Figure 1 as an example, the program generates a random four-base sequence to form *A*_*i*_, *B*_*i*_, #, *ψ*, *X* and *Y*, as shown in Table 5. Among them represents the ends of the DNA chains, *ψ* represents the vertex weight of the DNA string, *Y* and are used to represent the vertex and edge weight of the DNA string, then *A*_*i*_ and *B*_*i*_ are used to represent the vertex *v*_*i*_. So Table 6 shows the DNA node sequence composed by Braich's methods [41]. In the example mentioned in this paper, the DNA sequences of the six vertices are all shown in Table 6.

In the program, we generate random sequences to represent the initial data pool. The routes that meet the quota through the different vertices are shown in Table 7 (due to there are too many feasible solutions, we only show some of them). The optimal solution is derived from the composition structure of the last selected DNA sequences in Table 8. We can also obtain the best solution of the example from the running of the program. On the other hand, DNA computing algorithm is mainly based on the biological DNA molecular chemical reaction to achieve the output of the algorithm function. Because the computer programs are executed in sequence, it is impossible to realize the parallel chemical reaction operation of molecules in DNA algorithm. Therefore, the Python program designed by our simulation analysis can only realize the biological experiment results we designed. Compared with other algorithms (Ant colony algorithm [50], Particle Swarm Optimization algorithm [51], Genetic algorithm [52]), DNA algorithm is not ideal because of the different computing mechanism. However, as the technology for DNA experiments matures, the parallel advantages of DNA computing will be fully demonstrated.

## 5. Conclusions

The main result of the work is that the QTSP in an arbitrarily undirected graph can be solved using the Adleman-Lipton model. The process uses biological manipulation to produce combination results and screen out solutions. Through computer simulation, the design of DNA coding and the operations of the algorithm are completed. The proposed algorithm is based on DNA molecules, and has obvious advantages in terms of computing speed, storage capacity and energy consumption. So far, there are few methods to solve the QTSP. Considering the online traveling salesman problem, Ausiello et al. [11] presented the lower bounds of online QTSP and the competitive strategies in positive semi-axis and general network situations. Yu et al. [12] proposed an optimal deterministic algorithm for each variant defined in general space, solid line or half line. For QTSP with known city quota, our proposed algorithm will have a better advantage in computing efficiency with the increasing of problem scale. Because the computational complexity, experimental test tubes and chains length of our algorithm are all polynomial time complexity (Theorem 1 and 2). In the Adleman-Lipton model, every DNA manipulation used can be achieved through biochemical reactions in the laboratory. We take the problem with six points as an example, and obtain the optimal solution of QTSP through the Python program simulation. We believe that through the maturity of DNA experimental technology, the real results in the experimental environment will also be confirmed.

Currently, DNA computing algorithms for different complex problems are being proposed, for example, Wu et al. [48] and Tian et al. [31] used DNA computing to solve the family traveling salesperson problem and job shop scheduling problem respectively, achieving great efficiency gains in terms of algorithmic computational complexity. In addition, DNA computing has been increasingly applied to different scenarios, such as image recognition [53], artificial neural network design [54] and quantum computing [55]. It is foreseen that pioneering research in the cross-fertilisation of DNA computing with disciplinary needs will drive significant developments in many aspects of science and technology. The latest advances in DNA computing are shown in Table 9.

At present, DNA computing has unparalleled advantages in dealing with NP-hard problems, because traditional algorithms cannot effectively process large amounts of data. Meanwhile, existing data often suffers from uncertainty and inaccuracy. In such cases, parallel processing of data using the latest generation of technology seems to be useful [58]. The theoretical research and practical realization of DNA computing for many related problems that have not yet been solved are also the direction of our future research. How to combine DNA computing with other computing methods to solve the remaining NP problems still has further exploration. It will lead to further research and more challenging development in biotechnology. In addition, in the future we will focus on combining DNA computing with the latest deep learning models including attention mechanisms, as well as quantum computing, nanotechnology, so that the parallelism of the models can be fully exploited and DNA computing can be extended to a wider range of applications [59–62].

## Figures and Tables

**Figure 1:** DNA double helix structure.

**Figure 2:** The distance between vertices and the quota of vertices, respectively.

**Figure 3:** Flowchart for computing the QTSP.

**Algorithm 1:** Generate various routings strands.

**Algorithm 2:** Remove the chains representing routes that go through multiple vertices.

**Algorithm 3:** Add vertex weights to different paths.

**Algorithm 4:** Append edges weight chains.

**Algorithm 5:** Get the optimal solution strands.

**Table 1:** Notations and symbols.

Symbol	Description
*V*	Vertex set
*E*	Edge set
*w*_*i*_	Quota of the *i*-th vertex
*d*_*i*,*j*_	The distance between *i*-th vertex and *j*-th vertex
*A*_*i*_, *B*_*i*_	DNA string of the *i*-th vertex
*X*	DNA string representing weight
*n*	Number of vertices
*m*	Number of edges
*v*_*i*_	The *i*-th vertex
*Q*	Minimum quota for problems
#	Start and end flags of DNA strands
*Y*	DNA string representing vertex

**Table 2:** An example of the QTSP instance naming.

The PCTSP intance	*σ*	Suffix	The QTSP instance
problem_20_100_100_1000.pctsp	0.2	2	problem_20_100_100_1000_2.qtsp
	0.5	5	problem_20_100_100_1000_5.qtsp
	0.8	8	problem_20_100_100_1000_8.qtsp

**Table 3:** Results of the QTSP instances.

Id	Name	*n*	*Q*	*Q*_*r*_	*D*_*r*_	Time (s)
1	problem_20_100_100_1000_2.qtsp	20	154	181	294	0.1018
2	problem_20_100_100_10000_2.qtsp	20	187	215	2400	0.5031
3	problem_20_100_1000_1000_2.qtsp	20	179	215	330	0.101
4	problem_20_100_1000_10000_2.qtsp	20	168	199	4387	0.344
5	problem_20_100_10000_1000_2.qtsp	20	181	315	288	0.1029
6	problem_20_100_10000_10000_2.qtsp	20	138	140	3973	0.6124
7	problem_40_100_100_1000_2.qtsp	40	338	395	196	1.130
8	problem_40_100_100_10000_2.qtsp	40	328	420	1835	0.5252
9	problem_40_100_1000_1000_2.qtsp	40	312	341	222	1.413
10	problem_40_100_1000_10000_2.qtsp	40	376	391	1861	1.209
11	problem_40_100_10000_1000_2.qtsp	40	356	359	222	1.509
12	problem_40_100_10000_10000_2.qtsp	40	407	413	1751	0.7927
13	problem_60_100_100_1000_2.qtsp	60	540	583	161	1.996
14	problem_60_100_100_10000_2.qtsp	60	516	519	1689	7.119
15	problem_60_100_1000_1000_2.qtsp	60	576	612	115	1.279
16	problem_60_100_1000_10000_2.qtsp	60	523	596	2212	18.01
17	problem_60_100_10000_1000_2.qtsp	60	478	495	183	7.687
18	problem_60_100_10000_10000_2.qtsp	60	556	650	1722	5.864
19	problem_80_100_100_1000_2.qtsp	80	697	730	185	265.2
20	problem_80_100_100_10000_2.qtsp	80	779	787	1763	109.7
21	problem_80_100_1000_1000_2.qtsp	80	739	766	132	8.856
22	problem_80_100_1000_10000_2.qtsp	80	775	789	1046	1.573
23	problem_80_100_10000_1000_2.qtsp	80	688	688	204	204.5
24	problem_80_100_10000_10000_2.qtsp	80	776	788	1802	28.49
25	problem_100_100_1000_1000_2.qtsp	100	1021	1047	91	3.367
26	problem_100_100_1000_10000_2.qtsp	100	960	1057	944	7.195
27	problem_100_100_10000_1000_2.qtsp	100	961	1031	113	169.2
28	problem_100_100_10000_10000_2.qtsp	100	837	837	1261	21.30
29	problem_20_100_100_1000_5.qtsp	20	386	405	651	0.7524
30	problem_20_100_100_10000_5.qtsp	20	469	482	3867	0.176
31	problem_20_100_1000_1000_5.qtsp	20	449	477	571	0.361
32	problem_20_100_1000_10000_5.qtsp	20	422	445	8319	0.7272
33	problem_20_100_10000_1000_5.qtsp	20	452	464	419	0.1934
34	problem_20_100_10000_10000_5.qtsp	20	347	351	6374	0.2405
35	problem_40_100_100_1000_5.qtsp	40	846	855	358	1.897
36	problem_40_100_100_10000_5.qtsp	40	821	898	3447	5.922
37	problem_40_100_1000_1000_5.qtsp	40	780	832	444	5.036
38	problem_40_100_1000_10000_5.qtsp	40	940	940	3384	2.254
39	problem_40_100_10000_1000_5.qtsp	40	892	897	426	14.48
40	problem_40_100_10000_10000_5.qtsp	40	1019	1059	3475	1.677
41	problem_60_100_100_1000_5.qtsp	60	1351	1368	419	14.16
42	problem_60_100_100_10000_5.qtsp	60	1291	1300	4407	25.11
43	problem_60_100_1000_1000_5.qtsp	60	1440	1461	385	2.656
44	problem_60_100_1000_10000_5.qtsp	60	1308	1323	4536	2.678
45	problem_60_100_10000_1000_5.qtsp	60	1196	1200	385	2.407
46	problem_60_100_10000_10000_5.qtsp	60	1390	1392	3623	12.80
47	problem_20_100_100_1000_8.qtsp	20	617	619	1097	0.3255
48	problem_20_100_100_10000_8.qtsp	20	750	762	7565	0.2571
49	problem_20_100_1000_1000_8.qtsp	20	719	743	1045	0.311
50	problem_20_100_1000_10000_8.qtsp	20	675	691	14319	0.3447
51	problem_20_100_10000_1000_8.qtsp	20	724	728	774	0.2847
52	problem_20_100_10000_10000_8.qtsp	20	555	559	10480	0.516
53	problem_40_100_100_1000_8.qtsp	40	1354	1355	752	0.4747
54	problem_40_100_100_10000_8.qtsp	40	1314	1319	8439	12.23
55	problem_40_100_1000_1000_8.qtsp	40	1248	1251	782	8.271
56	problem_40_100_1000_10000_8.qtsp	40	1504	1507	6658	2.253
57	problem_40_100_10000_1000_8.qtsp	40	1427	1449	700	5.133
58	problem_40_100_10000_10000_8.qtsp	40	1630	1630	7850	2.513
59	problem_60_100_100_1000_8.qtsp	60	2161	2169	825	13.56
60	problem_60_100_100_10000_8.qtsp	60	2066	2074	8316	19.71
61	problem_60_100_1000_1000_8.qtsp	60	2304	2311	805	3.216
62	problem_60_100_1000_10000_8.qtsp	60	2093	2094	10206	72.78
63	problem_60_100_10000_1000_8.qtsp	60	1913	1927	810	3.029
64	problem_60_100_10000_10000_8.qtsp	60	2224	2228	8580	17.29

**Table 4:** Routes of the QTSP instances.

Id	Route
1	[0, 11, 8, 6, 15, 0]
2	[0, 13, 3, 16, 6, 12, 15, 0]
3	[0, 11, 2, 7, 8, 0]
4	[0, 14, 5, 15, 0]
5	[0, 8, 10, 19, 16, 0]
6	[0, 13, 15, 8, 16, 0]
7	[0, 12, 18, 5, 27, 20, 13, 17, 37, 0]
8	[0, 5, 12, 13, 39, 18, 32, 22, 0]
9	[0, 39, 36, 6, 25, 30, 27, 5, 0]
10	[0, 16, 36, 27, 19, 37, 3, 38, 31, 0]
11	[0, 6, 7, 37, 10, 30, 21, 0]
12	[0, 20, 13, 32, 21, 28, 25, 23, 17, 0]
13	[0, 45, 49, 59, 36, 51, 44, 54, 23, 18, 3, 0]
14	[0, 34, 3, 16, 8, 33, 55, 28, 39, 50, 0]
15	[0, 56, 50, 6, 19, 13, 7, 14, 10, 46, 43, 39, 36, 34, 41, 12, 55, 0]
16	[0, 30, 33, 39, 59, 43, 46, 15, 20, 42, 0]
17	[0, 14, 38, 25, 7, 57, 26, 31, 20, 21, 24, 46, 0]
18	[0, 32, 19, 4, 18, 57, 22, 34, 9, 59, 33, 0]
19	[0, 42, 70, 32, 13, 72, 19, 63, 78, 66, 58, 55, 41, 68, 0]
20	[0, 27, 56, 73, 55, 46, 77, 17, 67, 32, 9, 72, 11, 15, 60, 33, 0]
21	[0, 67, 72, 5, 55, 8, 17, 57, 70, 64, 63, 33, 52, 42, 38, 7, 51, 0]
22	[0, 44, 25, 28, 66, 29, 11, 52, 16, 75, 62, 46, 13, 51, 0]
23	[0, 59, 48, 34, 23, 40, 20, 41, 7, 50, 6, 5, 14, 78, 28, 47, 0]
24	[0, 10, 35, 15, 20, 79, 67, 26, 56, 60, 77, 70, 63, 30, 41, 0]
25	[0, 69, 70, 4, 32, 84, 93, 28, 41, 43, 31, 78, 91, 88, 2, 89, 17, 0]
26	[0, 17, 81, 55, 95, 99, 29, 71, 68, 94, 66, 22, 51, 16, 46, 2, 58, 79, 52, 30, 76, 75, 0]
27	[0, 69, 8, 11, 56, 49, 37, 25, 66, 89, 29, 44, 47, 53, 34, 59, 33, 96, 0]
28	[0, 42, 39, 21, 70, 33, 90, 78, 49, 51, 45, 97, 67, 17, 14, 91, 36, 60, 18, 3, 0]
29	[0, 15, 10, 9, 3, 14, 4, 11, 0]
30	[0, 15, 12, 6, 16, 3, 13, 17, 11, 18, 0]
31	[0, 11, 6, 14, 18, 7, 8, 17, 2, 12, 13, 0]
32	[0, 4, 7, 16, 19, 11, 14, 5, 15, 0]
33	[0, 4, 11, 1, 6, 3, 8, 10, 19, 16, 0]
34	[0, 13, 15, 11, 6, 18, 9, 4, 8, 16, 0]
35	[0, 12, 18, 5, 27, 20, 4, 10, 33, 1, 13, 35, 26, 22, 36, 31, 11, 29, 24, 37, 0]
36	[0, 22, 32, 6, 27, 38, 23, 16, 35, 1, 34, 3, 18, 37, 28, 10, 11, 12, 5, 0]
37	[0, 39, 36, 6, 25, 30, 17, 26, 37, 20, 38, 14, 13, 8, 23, 0]
38	[0, 16, 36, 21, 35, 38, 14, 34, 3, 37, 19, 7, 11, 24, 26, 15, 17, 31, 0]
39	[0, 21, 1, 17, 9, 8, 26, 7, 37, 10, 30, 3, 2, 31, 6, 0]
40	[0, 20, 13, 32, 39, 33, 14, 29, 4, 11, 38, 26, 3, 28, 25, 23, 17, 0]
41	[0, 45, 49, 59, 36, 56, 22, 18, 23, 54, 44, 51, 25, 14, 19, 34, 6, 42, 27, 50, 33, 37, 3, 0]
42	[0, 34, 1, 18, 5, 53, 58, 23, 10, 57, 14, 22, 48, 44, 52, 40, 30, 8, 33, 55, 28, 39, 50, 0]
43	[0, 55, 12, 30, 31, 48, 35, 20, 25, 42, 47, 43, 39, 36, 34, 41, 22, 23, 53, 57, 14, 7, 13, 19, 1, 17, 27, 50, 56, 0]
44	[0, 42, 20, 15, 3, 38, 37, 45, 52, 7, 22, 44, 17, 14, 55, 23, 40, 46, 43, 59, 39, 33, 30, 0]
45	[0, 46, 24, 21, 30, 48, 23, 54, 1, 39, 49, 7, 25, 47, 55, 11, 10, 33, 3, 53, 37, 35, 8, 20, 31, 26, 18, 0]
46	[0, 33, 59, 9, 34, 22, 57, 3, 11, 7, 20, 14, 24, 1, 41, 21, 50, 54, 56, 46, 53, 18, 4, 19, 32, 0]
47	[0, 11, 8, 9, 3, 14, 5, 17, 19, 7, 12, 16, 10, 15, 0]
48	[0, 13, 3, 16, 6, 1, 7, 9, 17, 11, 2, 18, 14, 15, 0]
49	[0, 13, 12, 2, 17, 8, 7, 18, 15, 9, 6, 16, 5, 4, 3, 11, 0]
50	[0, 4, 7, 12, 14, 11, 19, 16, 1, 3, 10, 13, 9, 2, 5, 15, 0]
51	[0, 8, 10, 19, 16, 12, 2, 11, 1, 6, 7, 15, 18, 4, 0]
52	[0, 16, 8, 4, 9, 18, 6, 11, 15, 13, 14, 5, 7, 12, 0]
53	[0, 37, 24, 29, 32, 6, 33, 10, 4, 20, 27, 9, 23, 11, 31, 34, 5, 38, 17, 13, 35, 26, 22, 36, 2, 30, 15, 18, 12, 0]
54	[0, 5, 2, 14, 4, 36, 25, 29, 32, 6, 27, 38, 23, 16, 35, 1, 34, 3, 18, 39, 37, 28, 10, 11, 12, 31, 9, 7, 33, 22, 0]
55	[0, 23, 25, 27, 30, 17, 26, 37, 24, 9, 1, 29, 4, 16, 22, 20, 38, 14, 13, 8, 2, 19, 33, 35, 21, 6, 36, 39, 0]
56	[0, 31, 18, 7, 19, 37, 3, 34, 30, 4, 29, 20, 1, 39, 26, 24, 11, 15, 17, 9, 22, 35, 21, 36, 16, 0]
57	[0, 18, 26, 7, 37, 10, 32, 20, 6, 31, 2, 3, 30, 39, 16, 33, 12, 1, 14, 38, 17, 9, 8, 27, 25, 29, 34, 21, 0]
58	[0, 20, 13, 27, 34, 19, 36, 6, 18, 10, 31, 37, 22, 2, 3, 26, 38, 11, 4, 29, 14, 33, 39, 32, 21, 28, 25, 23, 17, 0]
59	[0, 41, 8, 5, 53, 58, 24, 35, 11, 48, 38, 1, 39, 28, 33, 20, 37, 26, 55, 43, 10, 56, 22, 18, 23, 54, 44, 3, 50, 27, 42, 6, 34, 19, 14, 25, 51, 36, 59, 49, 45, 0]
60	[0, 34, 3, 26, 23, 58, 53, 5, 18, 1, 9, 16, 8, 30, 40, 52, 44, 41, 46, 49, 21, 59, 32, 56, 43, 48, 22, 14, 57, 10, 12, 20, 25, 27, 36, 51, 33, 55, 28, 39, 50, 0]
61	[0, 56, 50, 27, 13, 19, 1, 17, 24, 7, 14, 10, 46, 11, 32, 33, 30, 12, 55, 28, 54, 16, 43, 47, 42, 25, 20, 35, 48, 31, 41, 22, 5, 39, 36, 34, 8, 4, 59, 57, 53, 23, 26, 29, 58, 0]
62	[0, 42, 20, 15, 6, 51, 53, 44, 22, 7, 52, 45, 37, 38, 3, 10, 27, 48, 11, 2, 47, 36, 35, 16, 13, 8, 26, 25, 18, 49, 23, 50, 12, 17, 14, 55, 31, 40, 46, 43, 59, 39, 33, 30, 0]
63	[0, 46, 24, 21, 30, 29, 39, 49, 55, 47, 25, 7, 57, 38, 17, 32, 2, 58, 45, 27, 37, 53, 8, 35, 23, 42, 10, 33, 3, 16, 9, 12, 20, 31, 26, 18, 0]
64	[0, 32, 57, 3, 11, 7, 26, 45, 22, 34, 9, 38, 48, 8, 30, 28, 49, 16, 54, 50, 21, 41, 52, 25, 27, 37, 12, 2, 46, 53, 18, 4, 19, 58, 20, 14, 24, 1, 0]

**Table 5:** Sequences chosen to represent *A*_*i*_, *B*_*i*_, #, *ψ*, *X* and (*i* ∈ {1,2,…, 6}) for the QTSP in Figure 2.

Bit	3′ − 5′ DNA sequence	Bit	3′ − 5′ DNA sequence
*A*_1_	*GTTT*	*B*_1_	*GATG*
*A*_2_	*GTTA*	*B*_2_	*AGTT*
*A*_3_	*TACG*	*B*_3_	*ACTG*
*A*_4_	*GGAA*	*B*_4_	*GCGG*
*A*_5_	*TATT*	*B*_5_	*CTAG*
*A*_6_	*TCCC*	*B*_6_	*GCCG*
#	*GTAA*	*ψ*	*AGGC*
*X*	*CGAG*	*Y*	*TATA*

**Table 6:** Sequences chosen to represent the elements *A*_*i*_*B*_*i*_(*i* ∈ {1,2,…, 6}) for the QTSP in Figure 2.

Bit	3′ − 5′ DNA sequence	Bit	3′ − 5′ DNA sequence
*A*_1_ *B*_1_	*GTTTGATG*	*A*_2_ *B*_2_	*GTTAAGTT*
*A*_3_ *B*_3_	*TACGACTG*	*A*_4_ *B*_4_	*GGAAGCGG*
*A*_5_ *B*_5_	*TATTCTAG*	*A*_6_ *B*_6_	*TCCCGCCG*

**Table 7:** Routes and DNA strands satisfying quota through different vertices in Figure 2.

Routing	DNA strands
*v*_1_⟶*v*_2_⟶*v*_3_⟶*v*_6_⟶*v*_1_	3′ − *GTTTGATGGTTAAGTTTACGACTG*
	*TCCCGCCGGTTTGATG* − 5′
*v*_1_⟶*v*_2_⟶*v*_4_⟶*v*_5_⟶*v*_6_⟶*v*_1_	3′ − *GTTTGATGGTTAAGTTGGAAGCGG*
	*GTTTGATGGTTAAGTTGGAAGCGG* − 5′
*v*_1_⟶*v*_3_⟶*v*_5_⟶*v*_6_⟶*v*_1_	3′ − *GTTTGATGTACGACTGTATTCTAG*
	*TCCCGCCGGTTTGATG* − 5′
*v*_1_⟶*v*_3_⟶*v*_4_⟶*v*_5_⟶*v*_6_⟶*v*_1_	3′ − *GTTTGATGTACGACTGGGAAGCGG*
*v*_1_⟶*v*_3_⟶*v*_6_⟶*v*_2_⟶*v*_1_	3′ − *GTTTGATGTACGACTGTCCCGCCG*
	*GTTAAGTTGTTTGATG* − 5′
*v*_1_⟶*v*_4_⟶*v*_3_⟶*v*_6_⟶*v*_1_	3′ − *GTTTGATGGGAAGCGGTACGACTG*
	*TCCCGCCGGTTTGATG* − 5′
*v*_1_⟶*v*_5_⟶*v*_4_⟶*v*_3_⟶*v*_1_	3′ − *GTTTGATGTATTCTAGGGAAGCGG*
*v*_1_⟶*v*_6_⟶*v*_5_⟶*v*_4_⟶*v*_3_⟶*v*_1_	3′ − *GTTTGATGTCCCGCCGTATTCTAG*
	*GGAAGCGGTACGACTGGTTTGATG* − 5′

**Table 8:** DNA sequences chosen to represent the solutions to the QTSP in Figure 2.

Routing	DNA strands
*v*_1_⟶*v*_2_⟶*v*_5_⟶*v*_3_⟶*v*_1_	3′ − *GTTTGATGGTTAAGTTTATTCTAGTACGAC*
	*TGGTTTGATG* − 5′
*v*_1_⟶*v*_3_⟶*v*_5_⟶*v*_2_⟶*v*_1_	3′ - *GTTTGATGTACGACTGTATTCTAGGTTAAGTTGTTTGATG* − 5′

**Table 9:** Recent developments in DNA computing and their applications.

Scholars	Issues studied	Model name	Characteristics	Experimental results
Wu et al. [48]	Family traveling salesperson problem	Adleman-lipton model	*O*(*N*^2^) (*N* is the number of vertices in the problem without the origin)	Simulation of experimental benchmark examples, such as bruma14, ulysses16, ulysses22, eil51 and Berlin52 to demonstrate the feasibility of the algorithm

Roy et al. [53]	A robust image encryption framework	DNA computing and chaos theory	DNA computing helps to effectively encode the actual pixel values on which DNA operations can be applied	The proposed approach is tested on different types of images and the obtained results are very promising. On average, the proposed approach achieves approximately 96.95% of NPCR and 31.56% of UACI that is quite satisfactory

Mondal et al. [54]	Artificial neural networks and the implementation of DNA logic gates	Short DNA strands to develop artificial neural networks	Short sequences of DNA molecules can be used to encode input and output signals and to build the basic structure of a neuron. And using the secondary structure of DNA molecules to illustrate design strategies for logic gates	Qian et al. [56] propose a DNA gate architecture that uses a seesaw gate motif to develop linear threshold circuits. Cherry and Qian [57] developed artificial neural networks that can perform computational tasks, e.g. molecular pattern recognition, based on design guidelines for DNA circuits, i.e. predictable hybridisation rules for DNA strands and biochemical reactions

Chang et al. [55]	Independent set problem	Bio-molecular solutions on IBM quantum computers	They propose a bio-molecular algorithm with *O*(*n*^2^+*m*) biological operations, *O*(2^*n*^) DNA strands, (HTML translation failed) tubes and *O*(*n*) the longest DNA strand, for solving the independent set problem for any graph *G* with *m* edges and *n* vertices	A maximum independent set problem with three vertices and two edges is solved using the DNA computing algorithm and quantum circuits and correct results are obtained

Tian et al. [31]	Job shop scheduling problem	Adleman-lipton model	The DNA algorithm is proved to have an *O*(*n*^2^) complexity and the length of the final strand of the optimal schedule is within appropriate range	Experiment with 58 benchmark instances show that the proposed DNA algorithm outperforms other comparative heuristics

## Data Availability

The data used to support the findings of this study are included within the article.
